This article has been retracted.

# siRNA directed against c-Myc inhibits proliferation and downregulates human telomerase reverse transcriptase in human colon cancer Colo 320 cells

**DOI:** 10.1186/1756-9966-27-27

**Published:** 2008-08-12

**Authors:** Huang Hao, Yu Nancai, Fu Lei, Wei Xiong, Su Wen, Huang Guofu, Wu yanxia, Huang Hanju, Liu Qian, Xiao Hong

**Affiliations:** 1 Center of Experimental Medicine, Wuhan No.1 Hospital, Wuhan, 430022, PR China; 2 Department of Pathogentic Biology, Tongji Medical College, Huazhong University of Science and Technology, Wuhan, 430030, PR China; 3 Brain Research Center, University of British Columbia, Vancouver, BC, Canada

## Abstract

The c-Myc and human telomerase reverse transcriptase gene (hTERT) gene are frequently deregulated and overexpressed in malignancy. hTERT activity is induced by c-Myc and strategies designed to inhibit c-Myc expression in cancer cells may have considerable therapeutic value. We designed and used a short hairpin RNA to inhibit c-Myc expression in Colo 320 cells and validated its effect on cell proliferation. In this study, four c-Myc-shRNA expression vectors were constructed and introduced into Colo 320 cells. The effects of c-Myc silencing on tumor cell growth was assessed by soft agar assay and DNA synthesis experiments. The expressions of c-Myc and hTERT were also assessed by real-time reverse transcription-polymerase chain reaction and Western blot analysis. Upon transient transfection with plasmid encoding shRNA, it was found that expression of c-Myc and hTERT decreased in shRNA-transfected cells. The downregulation of c-Myc and hTERT inhibited cell growth, shortened telomere lengths, and suppressed telomerase activity. In conclusion, our findings demonstrate that shRNA of c-Myc can inhibit the DNA replication in Colo 320 cells effectively and reduce telomere length and telomerase activity, therefore, it could be used as a new potential anticancer tool for therapy of human colon cancer.

## Background

Telomerase is a ribonucleoprotein enzyme that synthesizes telomeres, i.e., DNA repeats that cap and protect the ends of chromosomes[1]. The core of the mammalian telomerase holoenzyme is the catalytic subunit, telomerase reverse transcriptase, which adds hexameric DNA repeats (TTAGGG) that correspond to the telomerase RNA component known as TERC[2,3]. Telomerase activation has been regarded as a crucial step in cellular carcinogenesis, and it is one of the most common molecular markers in a broad spectrum of malignancies [4]. It has been reported that telomerase activity is significantly high in about 80% of cancers and correlates well with the degree of malignancy[5]. Some studies have shown that hTERT gene expression is more specific and sensitive than telomerase activity in the diagnosis of malignant neoplasms, as the hTERT gene is overexpressed in about 90% of malignant tumors [6]. The control of c-Myc gene expression is a complex process and occurs at various steps of transcription, such as initiation, elongation, and attenuation, as well as during the post-transcriptional stages[7,8].

The protein product of the c-Myc protooncogene plays a vital role in the process of cellular growth and differentiation[9]. Deregulation of c-Myc expression has been detected in many cancers and is believed to be an important step in carcinogenesis [10]. In addition, c-Myc has also been implicated in the regulation of telomerase through its ability to induce the transcriptional activation of hTERT[11]. RNA interference (RNAi) has been described.

Recently, a post-transcriptional gene silencing pathway mediated by double-stranded RNA (dsRNA), also called RNA interference (RNAi) has been described[12,13]. RNAi is a natural mechanism of defence, which protects cells against exogenous dsRNA, such as viral or deriving from transposones[14]. When a dsRNA enters the cytoplasm, RNAse III Dicer can process it to produce several small interfering RNAs (siRNAs), 21–23 nucleotide long RNA molecules with 2 nucleotide long 3'overhangs. Small interfering RNAs may get incorporated into the RNA induced silencing complex (RISC), which identifies and silences complementary RNAs generally through a cleavage mechanism. In the last few years, it has been demonstrated that siRNAs represent an efficient tool to modulate the expression of a large number of cancer-related genes[15].

In the present study, we selectively downregulated c-Myc expression in human colon cancer Colo 320 cells with siRNA delivered via a plasmid-based polymerase III promoter system. This approach allowed us to explore a possible role for c-Myc in regulating telomerase activity.

## Methods

### Short-interfering RNA design

shRNA directed against c-Myc mRNA were selected using the computer program (web site ), and it was verified, by BLAST search, that there was no homology with another human gene. shRNA #1–4 sequences directed against c-Myc mRNA were selected according to Blast search score and GC content (40–60%). The shRNA expression cassette contained 19 nucleotide of the target sequence followed by the loop sequence (TTCAAGACG), reverse complement to the 19 nucleotide, stop codon for U6 promoter and BamHI site (c-Myc -1: 5'-CTATGACCTCGACTACGACTTCAAGACCGTCCTAGTCGAGGTCATAG-3'; c-Myc -2: 5'-AAATTCGAGCTGCTGCCC TTCAAGACG GGGCAGCAGCTCGAATTTC-3'; c-Myc -3: 5'GCCCCCAAGC TAGTTATC TTCAAGACG GATAACTACCTTGGGGGCC-3'; c-Myc -4: 5'CCACAGCATACATCCTGT TTCAAGACG ACAGGATGTATGCTGTGGC-3'). The shRNA cassettes and their complementary strands were synthesized (Wuhan Genesil Biotechnology, Wuhan, China).

### Cell culture and transfection

The colon cancer cell line Colo 320 was obtained from China Center for TypeCulture Collection (GDC298). The cells were grown in RPMI-1640 medium (GIBCO, Invitrogen, Carlsbad, CA) supplemented with 10% fetal bovine serum (Gibco BRL), 50 units/ml penicillin, and 50 μg/ml streptomycin. The Colo 320 cells were maintained in a humidified 37°C incubator with 5% CO_2_, fed every 3 days with complete medium, and subcultured when confluence was reached. The cells were routinely passaged every 1 or 2 days. For transfection, 2 × 10^5 ^cells were seeded into each well of a six well tissue culture plate (Costar). The next day (when the cells were 70–80% confluent), the culture medium was aspirated and the cell monolayer was washed with pre-warmed sterile phosphate-buffered saline (PBS). Cells were transfected with the pGensil-c-Myc -1, -2, 3, and -4 harboring green pEGFP-C1 green fluorescence protein reporter gene by using Lipofectamine 2000 reagent (Invitrogen, Carlsbad, CA) in accordance with the manufacturer's protocol. Cells were continuously cultured until harvest for analysis.

### Cell counts

Colo 320 cells were trypsinized on the indicated days and counted with a hemocytometer. We quantify cell proliferation by comparing the number of cells counted before and after transfection. Colo 320 Approximately 200 cells were evaluated in each sample using the hemocytometer. cell viability was assessed by trypan blue exclusion (Sigma-Aldrich China Inc, Shanghai, China).

### DNA synthesis

Colo 320 cells were treated with 1 mCi of 3H-thymidine per milliliter (Amersham Biosciences, Piscataway, NJ) for the last 6 h of day 3 after shRNA treatment. Cells were then rinsed twice with PBS, ice-cold 5% trichloroacetic acid, and 80% ethanol; the incorporated radioactivity of cell lysates was measured in a liquid scintillation counter.

### Soft agar colony assay

Two days after transfection, Colo 320 cells (300 cells per well) transfected with indicated plasmids were mixed with tissue culture medium containing 0.7% agar to result in a final agar concentration of 0.35%. Then 1 ml sample of this cell suspension was immediately plated in six-well plates coated with 0.6% agar in tissue culture medium (2 ml per well) and cultured at 37°C with 5% CO_2_. After 2 weeks, the top layer of the culture was stained with 0.2% piodonitrotetrazolium violet (Sigma). The culture was analyzed in triplicate, and colonies larger than 100 μm in diameter were counted.

### Quantification of c-Myc and hTERT mRNA

For the sqRT-PCR analysis, total RNA was isolated using Trizol reagent (Sigma) and reversely transcribed using random hexamers with Superscript II (Invitrogen). For c-Myc and hTERT detection, cDNA was mixed with the PCR reaction mixture and each c-Myc and hTERT-specific primer (LT5 and LT6). The PCR cycle number was set up to permit the distinction between mRNA expression profiles among the samples. PCR products were visualized on 1.2% agarose gel. Actin was used as an internal control, and positive and negative controls were always included. PCR reagents were from the Master Taq kit (Eppendorf).

### Telomere length measurement

Determination of telomere length was performed by Southern analysis of telomere restriction fragment (TRF) length. Genomic DNA was isolated from transfected cells using DNA isolation kit (Qiagen, Valencia, CA, USA) and quantified by UV spectrophotometry. Two micrograms of DNA were digested with restriction endonucleases RsaI and HinfI. The DNA digests were electrophoresed through 0.8% agarose and transferred to nylon membranes by capillary transfer in 20 × SSC as described.

After UV crosslinking (1200 μJ), the membranes were hybridized with a 3'-digoxigenin oligonucleotide probe with the sequence (CCCTAA)3'. After washing to remove unbound probe, an alkaline phosphatase-conjugated anti-digoxigenin antibody (Roche Applied Science, Indianapolis, IN, USA) was used for immunodetection of bound probe, followed by CDP Star chemiluminescence substrate (Roche Applied Science). Blots were exposed to X-ray film for 10–60 s. Mean TRF length and percentage photo-stimulated luminescence were determined from densitometric analysis of digital images of exposed films as described. Measurements of TRF length were performed in duplicate for each membrane.

### Detection of telomerase activity

The telomerase activity was measured using a PCR-TRAP ELISA kit (Roche, USA) according to the manufacturer's description with some modifications. For the TRAP reaction, 2 μg total RNA was added to 25 μl of reaction mixture with the appropriate amount of sterile water to create a final volume of 50 μl. Hybridization and the ELISA reaction were carried out following the manufacturer's instructions.

### Western blotting

Transfected cells were washed twice with PBS and suspended in IPH lysis buffer (50 mM Tris (pH 8.0), 150 mM NaCl, 5 mM EDTA, 0.5% NP40, 100 mM phenylmethyl sulfonyl fluoride leupeptin 1 mg/mL, aprotinin 1 mg/mL, and 1 M dithiothreitol). Cells were extracted at 4°C for 30 min. After centrifugation at 12,000 rpm for 20 min, the supernatant was subject to electrophoresis on 10% sodium dodecyl sulfate-polyacrylamide gel (SDS-PAGE), and transferred to a polyvinylidene difluoride (PVDF) membrane. The membrane was allowed to react with anti-β-actin polyclonal, anti-c-Myc and hTERT antibody (Santa Cruz Biotechnology). Specific antibodies were detected with a chemiluminescence kit (Sigma Life Science) according to the supplier's manual. Chemiluminescence was detected by exposure to X-ray film.

### Statistical analysis

All data in the text and figures is presented as means ± standard deviation (means ± SD). Statistical analysis was performed using Student's t-test.

## Results

### Effect of the c-Myc small interfering RNA on cell growth

As the first step, transfection efficiency of the plasmid encoding shRNA for c-Myc in Colo 320 cells was examined by coexpressing pEGFP green fluorescence protein. When the cells were examined under a fluorescence microscope 24 h after transfection, more than 75–85% of them was transfected (Figure 1A).

We then tested whether RNAi-mediated c-Myc could influence the ability of Colo 320 cells to form colonies in soft agar. Colo 320 cells were transfected with pGensil-c-Myc or empty vector. At 48 hours after transfection, the cells were placed into medium with soft agar, and colonies were counted after 2 weeks. RNAi directed against c-Myc resulted in a significant decrease (about 65%) in colony formation in Colo 320 cells (Figure 1B-1,2,3). These results showed that suppression of c-Myc by RNAi could decrease the ability of colon cancer cells to form colonies in soft agar.

Since four constructs gave similar results, we describe the results with pGenesil – c-Myc -1 in the subsequent experiments. We also evaluated the effect of c-Myc-specific shRNA on Colo 320 cell proliferation. Cell proliferation was measured by counting the number of viable cells using trypan blue staining. Transfected c-Myc-shRNA (Figure 1C-1) resulted in a marked inhibition of cell proliferation over this 2-day period and the shRNAs induced anti-proliferative effect was dose dependent. Cell growth was not influenced significantly by treatment with control-shRNA and vector. The statistical analysis shows that Colo 320 cell proliferation was affected by silencing of c-Myc. This is further confirmed with DNA synthesis assay using 3H-thymidine. In Figure 1C-2, the cell control and vector showed the maximum counts of (3H) thymidine (around 1400 and 1350 cpm/μgDNA) when compared to the treatment groups. In addition, the anti-proliferative effect was dose dependent and maximum inhibition was achieved with 12.5 μM shRNA.

**Figure 1:** **Effect of shRNA on proliferation of Colo 320 cells**. A. Plasmid pGenesil-c-Myc-1,-2, -3, and -4 with pEGFP encoding green fluorescence protein were transfected to the cells. B. c-Myc-depletion inhibits colony formation of Colo 320 cells. B-1) Control Colo 320 cells. B-2) Colo 320 cells treated with pGenesil-c-Myc-1 for 24 h B-3) The percentage of colonies of pGenesil-c-Myc-1 treated cells standardized against the corresponding control. C. Cells were treated with increasing concentrations of shRNA for 48 h. C-1)Cell viability was determined by cell counts. Results are expressed as the percentage of viable cells in the treatment groups with respect to that in the corresponding control. C-2) Cell proliferation following shRNA treatments for 48 h was quantified by 3H-thymidine incorporation studies. All data were obtained from three independent experiments. Error bars represent means ± SEM. Significantly different from the corresponding control (**P < 0.01, vs control. ##P < 0.01, vs vector).

### Down-regulation of c-Myc and hTERT by expression of shRNA

Compared with untreated cells, c-Myc and hTERT mRNA abundance was significantly decreased in cells incubated with 5, 7.5, 10, or 12.5 μM shRNA for 48 h (P < 0.01). Control and empty vector group markedly expressed c-Myc mRNA (Figure 2A) (P < 0.01).

**Figure 2:** **Effect of shRNA on expression of c-Myc and hTERT gene in Colo 320 cells**. A. c-Myc and hTERT mRNA expression of Colo 320 cells was detected by RT-PCR with different treatments. The cells were subjected to no treatment (control), pGenesil-vector group, 5, 7.5, 10, 12.5 μM shRNA for 48 h. B. c-Myc protein and hTERT expression of Colo 320 cells was detected by Western blotting with different treatments. Typical Western blot results for c-Myc and hTERT protein. Protein expression of c-Myc in Colo 320 cells was quantified by densitometric analysis. All data were obtained from three independent experiments. Error bars represent means ± SEM. Significantly different from the corresponding control (**P < 0.01, vs control. ##P < 0.01, vs vector).

As Western blot analysis indicated, the shRNA was able to reduce c-Myc and hTERT protein expression. As indicated in (Figure 2B), shRNA treatment inhibited the protein expression levels of c-Myc genes, representative downstream targets for c-Myc and hTERT protein in Colo 320 cells (P < 0.01). Transfection with shRNA at different concentrations (0, 5,7.5, 10, 12.5) resulted in the significant attenuation of expression of c-Myc and hTERT protein (P < 0.01). In contrast, β-actin protein expression was not affected by shRNA. These data indicated that vector-based RNAi could effectively suppress c-Myc and hTERT over-expression.

### Effects of shRNA on telomere length and telomerase activity

We evaluated the effect of shRNA on telomerase activity. Our data suggested that shRNA could down-regulate telomerase activity in shRNA-transfected groups. Telomerase activity were shown in Figure 3A. It revealed that shRNA-transfected groups had lower telomerase activity than the control groups. shRNA at a variety of concentrations resulted in significant reduction of telomerase activity.

**Figure 3:** **Effects of shRNA on telomere length and telomerase activity in Colo 320 cells**. A. Representative the concentration-course analysis of telomerase activity, each groups cells were mixed with 1 ml TBA solution for preparation of protein extract and 1 μg protein was subjected to TRAP assay. After hybridization and ELISA procedure, the absorbance of the samples at 450 nm was measured. The cells were subjected to no treatment (control), pGenesil-vector group, 5, 7.5, 10, 12.5 μM shRNA for 48 h. B. Mean telomere restriction fragment length was detected by RT-PCR with different treatments by Southern analysis as described under Materials and methods. Typical Southern blot results for telomere restriction fragments. Locations of the base pair markers on the DNA ladder are indicated along the left side. Significant difference was observed between the mean telomere lengths of the control and shRNA-transfected groups cells. All data were obtained from three independent experiments. Error bars represent means ± SEM. Significantly different from the corresponding control (**P < 0.01, vs control. ##P < 0.01, vs vector).

TRF length then was determined using pulse gel electrophoresis followed by Southern blot hybridization with telomere-specific probes. Average telomere length is shown in Figure 3B-1. Telomere length in shRNA-transfected groups telomeres was shorter than the one in the control groups. Transfection of shRNA resulted in significant increment of mean telomere length (Figure 3B-2, P < 0.05).

## Discussion

Some researchers have shown that c-Myc act as a transcription factor, which binds with E-box sites (CACGTG) of a gene's *cis*-element to regulate other gene transcription, such as hTERT gene[16]. C-Myc forms a dimer with Max, then binds to the specific E-box site sequence 5'-CACGTG-3' to transactivate target genes[17]. In contrast, c-Myc may also form a dimer with mad1 at the same binding site to suppress the transcription of target genes[18].

It has been shown that telomerase is highly related with malignant neoplasms [19]. When cells change from the normal growth status to abnormal growth status, there is persistent telomerase activity[20]. Previous studies showed that hTERT expression is related to many factors; in particular, that hTERT transcript regulation is affected by different transcription factors such as c-Myc[21,22]. Others report that activation or inhibition of c-Myc expression can change hTERT promoter activity[23,24]. The up-regulation, of c-Myc can *trans*-activate hTERT promoter and consequently activates telomerase. Xu *et al *suggest that c-Myc can activate hTERT transcription in a dose-dependent manner in leukemia cells. Several studies have shown that downregulating c-Myc activity induces tumor shrinkage[25].

In the present study, we used vector-based shRNA technique and constructed the recombinant plasmid expressing c-Myc-shRNA to transfect Colo 320 cells. Our results demonstrated that a transient reduction of c-Myc protein level by RNAi could significantly inhibit the growth rate of Colo 320 cells and its ability to form colonies in soft agar. Based on the results of western blotting, we also confirmed that the specific c-Myc-shRNA designed and used in this study successfully reduce the expression of the c-Myc and hTERT. We also found the We also found the attenuation of c-Myc and hTERT protein expression was dose-dependent.

Telomerase activity is strongly associated with telomere length maintenance. In the present study, we analyzed telomere length and telomerase activity in shRNA-transfected Colo 320 cells. Fig. 3 shows that the shRNA-transfected group had a shorter telomere length and lower telomerase activity than control group. Therefore, shRNA can significantly reduce telomere length and telomerase activity in siRNA-transfected Colo 320 cells.

In summary, we have identified the c-Myc shRNA that specifically inhibits activated c-Myc and suppresses cell proliferation. The c-Myc shRNA is able to block c-Myc DNA-binding activity and reduces the levels of c-Myc mRNA. Meanwhile, c-Myc shRNA can significantly reduce telomere length and telomerase activity in shRNA-transfected Colo 320 cells. Targeting c-Myc activation with RNAi may hold therapeutic promise for colon cancer with c-Myc and telomerase activation.
